# Research on Human Sports Rehabilitation Design Based on Object-Oriented Technology

**DOI:** 10.1155/2021/6626957

**Published:** 2021-03-04

**Authors:** Dandan Cao, Junyan Wang, Naihong Liu

**Affiliations:** Taiyuan University of Science and Technology, Taiyuan 030024, China

## Abstract

In order to improve the effect of human motion rehabilitation, a design model of human motion rehabilitation based on object-oriented technology is proposed. The entire model design process includes the following steps. First, a visual dynamic tracking model for human motion rehabilitation is established, and then a fuzzy PID (Proportion Integration Differentiation) superheterodyne control method is used to design the bone training control for human motion rehabilitation. The bone tracking control and adaptive training are under the control of object-oriented technology; it is analyzed by collecting human activity data during training. The 6-DOF kinematics problem of human movement rehabilitation is decomposed into the bone training control problem in the subspace. Combining object-oriented technology, visual blur recognition of human sports rehabilitation training, and adopting an adaptive kinematics model to design sports rehabilitation can improve the control convergence and global stability of the human sports rehabilitation process. The simulation results show that the method has a good overall steady state and the sports rehabilitation training effect is obvious.

## 1. Introduction

With the improvement of sports infrastructure and the development of sports, Chinese sports enthusiasm has been improved. However, in the process of rehabilitation training for injuries caused by various accidental conditions, the rehabilitation cycle of sports injuries is long due to the lack of systematic theoretical guidance and the corresponding knowledge base and it is easy to cause adverse physical injury sequelae. In order to promote the development of sports, it is necessary to systematize the theory of sports rehabilitation training. People do not know enough about sports injuries due to various accidents, especially the lack of systematic exercise rehabilitation training guidance; it is easy to cause the rehabilitation cycle to be too long and even leave the danger of the sequelae of physical injury [1]. Especially for students in school, the lively nature of young people makes them too keen on high-load sports such as football, basketball, boxing, and so on, which may cause a series of physical injuries in the process of exercise. There are many possibilities for sports injury, especially for the daily exercise of students in school at present, the main reasons are overload exercise, non-standard exercise methods and inadequate sports protection. Especially for high-intensity sports, such as basketball, football, and boxing, young people's excessive passion can easily cause physical damage in the process of release, such as wear, dislocation, viscera damage, and so on [2].

Rehabilitation training for physical injury has become the consensus of sports protection. This is mainly due to the fact that a large number of practices have proved that the traditional “bed rest” method for sports injury cannot complete the rehabilitation effect of sports injury, or cause the recovery of sports injury to be slower [3]. The body will leave sequelae during rest, which will affect the body's functions. However, there are many problems in sports rehabilitation training, mainly due to the imperfection of its sports rehabilitation training system and the lack of basic theoretical knowledge of corresponding sports rehabilitation training, such as overload and discontinuity in its practical use. Lack of systematicness, poor pertinence, and too much dependence on objective requirements lead to poor effect of sports rehabilitation training and even secondary damage to body function. Therefore, some systematic principles should be followed in the exercise rehabilitation training [4].

The design process of human motion rehabilitation is an object-oriented control process. The control of human body motion rehabilitation and human-machine motion planning are typical motion planning problems with multiple constraints in high-dimensional C-space. In order to improve the effect of human sports rehabilitation, this paper presents a design model of human sports rehabilitation based on object-oriented technology and constructs a visual dynamic tracking model of human sports rehabilitation [5]. The fuzzy PID hyperheterodyne control method is used to design the bone training control of human body movement rehabilitation, and the bone tracking control and adaptive training are carried out under the control of object-oriented technology [6]. The 6-DOF (degree of freedom) kinematics problem of human motion rehabilitation is decomposed into the skeletal training control problem in subspace, and the visual fuzzy recognition of human sports rehabilitation training is realized by combining the object-oriented technology. Adaptive kinematics model is used to design sports rehabilitation to improve the control convergence and global stability of human sports rehabilitation. Finally, the simulation results show the effectiveness of this method in improving the control stability of human sports rehabilitation process [7].

The research contributions of the thesis mainly include the following:

1. A design model of human motion rehabilitation based on object-oriented technology is proposed
2. Fuzzy PID (proportional integral derivative) superheterodyne control method is used to design the bone training control system for human movement rehabilitation
3. Combining object-oriented technology, visual blur recognition of human sports rehabilitation training, and adopting adaptive kinematics model to design sports rehabilitation

The rest of this paper is organized as follows.  Section 2 discusses kinematics model of human sports rehabilitation and control constraint parameter analysis, followed by the control model optimization discussed in Section 3. Simulation experiment and result analysis are discussed in Section 4.  Section 5 concludes the paper with summary and future research directions.

## 2. Kinematics Model of Human Sports Rehabilitation and Control Constraint Parameter Analysis

### 2.1. Skeletal System Modeling

When the man-machine system model was established in the AnyBody, the complexity of the organization was negatively correlated with the efficiency of the operation. The organization model should be simplified as much as possible. The exoskeleton model is simplified as a form in which a plurality of rods are connected. The length of the rods is a fixed length and corresponds to the body segment parameters of the experimental subject, and a pedal is added to the exoskeleton to drive the ankle joint movement [8]. Draw a simplified 3D model and import it into AnyBody in STL format. Because the simulation mainly analyzes the muscle-related parameters of the lower extremities as the object of study, in order to improve the speed of operation, when setting up the mannequin, the upper extremity ignores and removes most of the trunk muscles. Adjust the initial position of the human model to contact the exoskeleton model. With AnyBody's criteria for degrees of freedom and constraints to adjust the connection between the human model and the exoskeleton model, it is connected in a manner close to the real situation [9]. The original skeletal system model and the improved skeletal system model are shown in Figures 1 and 2.

It can be seen from Figures 1 and 2 that the establishment of a simplified 3D model can well simulate the motion parameters of human body, which has a good guiding significance for the subsequent collection of human motion data.

### 2.2. Kinematics Model of Human Sports Rehabilitation

Visual dynamic tracking model of human sports rehabilitation is built, and the kinematics model of human sports rehabilitation is established [10]. This paper assumes that the longitudinal movement of human body sport rehabilitation training process is symmetrical, and that the longitudinal movement is symmetrical in the process of longitudinal movement, in which the object-oriented technology is used to optimize the control design of human sports rehabilitation training [11]. The tilt control mechanism and the yaw operation mechanism of human body movement rehabilitation have no action. Given the initial configuration of human sports rehabilitation training model ***θ***_start_ ∈ **C**_free_ (free C- space), object pose **p**_obj_, and feasible grab set **g**_*c*_, let the movement chain of human sports rehabilitation training model composed of waist and left (right) arm be described as {*A*^0^, *A*^1^}; the homogeneous matrix ^*i* − 1^**T**_*i*_(*q*_*i*_) between i-1 and i-1 can be expressed as [12]

(1) Tii−1qi=ci−cαisisαisiaicisicαicisαiciaisi0sαicαidi0001.

The equations of longitudinal motion for human sports rehabilitation are obtained as follows:

(2) $$\begin{array}{c} m\frac{\text{d}V}{\text{d}t}=P\;\cos\;\alpha -X-mg\;\sin\;\theta , \end{array}$$

(3) $$\begin{array}{c} mV\frac{\text{d}\theta }{\text{d}t}=P\;\sin\;\alpha +Y-mg\;\cos\;\theta , \end{array}$$

(4) $$\begin{array}{c} J_{z}\frac{\text{d}\omega_{z}}{\text{d}t}+\left(J_{y}-J_{x}\right)\omega_{y}\omega_{x}+J_{xy}\left(\omega_{y}^{2}-\omega_{x}^{2}\right)=M_{z}, \end{array}$$

(5) $$\begin{array}{c} \frac{\text{d}x}{\text{d}t}=V\;\cos\;\theta , \end{array}$$

(6) $$\begin{array}{c} \frac{\text{d}y}{\text{d}t}=V\;\sin\;\theta , \end{array}$$

(7) $$\begin{array}{c} \frac{\text{d}\vartheta }{\text{d}t}=\omega_{z}, \end{array}$$

(8) $$\begin{array}{c} \alpha =\vartheta -\theta , \end{array}$$

(9) $$\begin{array}{c} \delta_{z}=f\left(e_{1}\right). \end{array}$$

Here, *x*, *y* are the position of centers of mass, *ω*_*x*_, *ω*_*y*_ indicate that the angular velocity of *XOY* axis in the body coordinate system *Ox*_1_, *Oy*_1_ mean the pitch angle of rehabilitation of human body, *δ*_*z*_ means the error of control system, and the quality of human body is indicated by the error of the control system and the error of the control system is indicated by the position of center of mass. C indicates the resistance, lift, and lateral force acting on the human body for rehabilitation training, in which the waist *X*, *Y* are regarded as the root of the movement chain, and the forward kinematics equation of the right arm of the human body can be used for intelligent feature extraction by the right hand. It includes six degrees of freedom of rotation, such as deflection angle *α*_0_, pitch angle *β*_0_, and rolling angle *β*_0_, which describe the motion of waist joint [13]. A six-degree-of-freedom control model of human sports rehabilitation training is constructed, which can be expressed as follows:

(10) $$\begin{array}{c} q_{0}={\left[\alpha_{0},\beta_{0},\gamma_{0}\right]}^{T}\equiv {\left[\theta_{1},\theta_{2},\theta_{3}\right]}^{T}. \end{array}$$

It can be seen that the longitudinal motion equation of human exercise rehabilitation training model is a group of dynamic systems composed of nonlinear differential equations. The elbow joint center of human sports rehabilitation training model is driven by mechanics through the wrist joint. The present kinematics model is constructed [14].

### 2.3. Analysis of Control Constraint Parameters for Human Sports Rehabilitation

Given the initial configuration of human sports rehabilitation training model ***θ***_start_ ∈ **C**_free_ (free C-space), pose **p**_obj_ of objects, and feasible grab set **g**_*c*_, the equations corresponding to the elements of both sides of the two matrices of human sports rehabilitation around the arm can be solved as [15]

(11) $$\begin{array}{c} q_{5}\equiv \theta_{8}=a\;\tan\;2\left(\pm o_{ey},\pm o_{ex}\right), \end{array}$$

(12) $$\begin{array}{c} q_{6}\equiv \theta_{9}=a\;\tan\;2\left(-o_{ez},-c_{5}o_{ex}-s_{5}o_{ey}\right), \end{array}$$

(13) $$\begin{array}{c} q_{7}\equiv \theta_{10}=a\;\tan\;2\left(-s_{5}n_{ex}+c_{5}n_{ey},s_{5}a_{ex}-c_{5}a_{ey}\right). \end{array}$$

This paper deduces the analytical form of inverse kinematics of arm in the model of human exercise rehabilitation training and obtains six rotational degrees of freedom of the left (or right) arm *A*^1^ including shoulder, elbow, and wrist, which are expressed as **q**_1_=[*q*_1_,…,*q*_7_]^*T*^ ≡ [***θ***_4_,…,***θ***_10_]^*T*^, and then obtains the exercise rehabilitation training of human body. The IK analytic equation of model control is used to realize the sixth-degree control model design of rehabilitation human sports rehabilitation training model. Combined with kinematics model [16], the constraint parameter model of skeletal training control for human exercise rehabilitation is constructed as follows:

(14) $$\begin{array}{c} \frac{\partial L}{\partial C_{i}}=2MC_{i}+\eta 1, \end{array}$$

where *M*=*λS*_*i*_^*T*^*S*_*i*_+(*X*_*i*_ − *D*_*i*_)^*T*^(*X*_*i*_ − *D*_*i*_)+***θ****I*.

In order to find the extremum, set ∂*L*/∂*C*_*i*_=0; then

(15) $$\begin{array}{c} C_{i}=-\frac{1}{2}\eta M^{-1}1. \end{array}$$

Based on the object-oriented technology, the machine vision tracking recognition method is used to recognize the dynamic process of rehabilitation, and the visual dynamic tracking model of human body movement rehabilitation is constructed to improve the dynamic control ability of rehabilitation training [17].

## 3. Control Model Optimization

### 3.1. Control Design of Bone Training for Human Body Movement Rehabilitation

The fuzzy PID superheterodyne control method is used to design the bone training control of human body movement rehabilitation, the bone tracking control and adaptive training of human body movement rehabilitation are carried out under the control of object-oriented technology, and the human body movement rehabilitation training is carried out [18]. The equivalent control law of model control is

(16) $$\begin{array}{c} u_{\text{eqx}}=\frac{\lambda \left(-\overset{\wedge }{f_{x}}-\lambda_{x}{\dot{e}}_{x}-\alpha e_{x}+\overset{..}{x}\right)}{\left(\lambda g_{x}+g_{\theta }\right)}. \end{array}$$

Some parameters of the control system of human sports rehabilitation training model are measured, and then the model is modified according to the measurement [19]. Several constraints of the model system are obtained as follows:

(17) $$\begin{array}{c} X_{\text{RL}}=R\times \theta_{\text{RL}}, \end{array}$$

(18) $$\begin{array}{c} X_{\text{RR}}=R\times \theta_{\text{RR}}, \end{array}$$

(19) $$\begin{array}{c} X_{\text{RL}}-X_{\text{RR}}=D\times \delta , \end{array}$$

(20) $$\begin{array}{c} {\dot{X}}_{P}={\dot{\theta }}_{P}L\;\cos\;\theta_{P}+{\dot{X}}_{\text{RM}}, \end{array}$$

(21) $$\begin{array}{c} Y_{P}=L\;\cos\;\theta_{P}, \end{array}$$

(22) $$\begin{array}{c} {\dot{Y}}_{P}=-{\dot{\theta }}_{P}L\;\sin\;\theta_{P}, \end{array}$$

(23) $$\begin{array}{c} X_{\text{RR}}+X_{\text{RL}}=2X_{\text{RM}}. \end{array}$$

In order to eliminate the effect of parameter estimation on the stability of skeletal training for human exercise rehabilitation, the third Lyapunov function is chosen as follows:

(24) $$\begin{array}{c} V_{3}=V_{2}+\frac{\lambda_{1}\zeta_{1}^{2}}{2}+\frac{\lambda_{2}\zeta_{2}^{2}}{2}+\frac{{\tilde{\delta }}^{2}}{2\varepsilon_{1}\delta }. \end{array}$$

In order to obtain the desired stability characteristics, the skeleton training process of human motion rehabilitation is controlled [20], and the nonlinear integral substitution control law is designed to limit the steady-state prediction error:

(25) $$\begin{array}{c} u=u_{eqx}+u_{eq\theta }+u_{sw}. \end{array}$$

The inverse kinematics problem of 6-DOF human exercise rehabilitation is decomposed into two sub-inverse kinematics problems with smaller dimensions. The adaptive regulation of skeletal training for human sports rehabilitation is chosen as follows:

(26) $$\begin{array}{c} V_{1}=\frac{1}{2}e_{1}^{2}. \end{array}$$

The derivation of the Lyapunov function for the skeletal training of human sports rehabilitation is

(27) $$\begin{array}{c} {\dot{V}}_{1}=e_{1}e_{2}-c_{1}e_{1}{}^{2}-e_{1}\lambda_{1}\zeta_{1}. \end{array}$$

By using the inverse design method and the combination of fuzzy control and adaptive control, the corresponding Lyapunov function is found and the derivative is obtained [21]:

(28) $$\begin{array}{c} {\dot{e}}_{2}={\dot{\omega }}_{2}-{\dot{\omega }}_{2r}, \end{array}$$

(29) $$\begin{array}{c} e_{2}=\alpha V^{2}+mg\left(\sin\;\vartheta +V\omega_{2}\right)+m\left(\cos\;\vartheta +V\omega_{2}\right)+c_{1}e_{2}+\lambda_{1}e_{1}-c_{1}^{2}e_{2}-c_{1}\lambda_{1}\zeta_{1}-{\ddot{\vartheta }}_{r}. \end{array}$$

### 3.2. Process Control Design of Rehabilitation Training

The control function of the mechanical tracking controller for human sports rehabilitation training is obtained as follows:

(30) $$\begin{array}{c} V_{2}=V_{1}+\frac{1}{2}e_{2}^{2}. \end{array}$$

Derivative:

(31) $$\begin{array}{c} {\dot{V}}_{2}={\dot{V}}_{1}+e_{1}{\dot{e}}_{2}. \end{array}$$

The inverse kinematics problem of 7-DOF right arm is decomposed and the control model of two degrees of freedom is obtained. The total degrees of freedom of skeletal training for human sports rehabilitation are 10. The configuration of human rehabilitation training can be expressed as ***θ***=[**q**_0_^*T*^, **q**_1_^*T*^]^*T*^ ≡ [***θ***_1_,…,***θ***_10_]^*T*^. Set $q_{1}={\left[\begin{array}{ccc} q_{1}, & \ldots , & q_{7} \end{array}\right]}^{T}$.sin *q*_*i*_ and cos *q*_*i*_ recorded as *s*_*q*_*i*__ and *c*_*q*_*i*__, respectively. The initial motion mechanics error compensation of the human body movement rehabilitation training model is *S* and the body posture error compensation of the training is ***θ***_start_=[***θ***_1start_,…,***θ***_10start_]^*T*^.

The design of control error compensation based on Lyapunov method is realized. According to Barbalat's theorem,

(32) $$\begin{array}{c} \underset{t⟶\infty }{\lim}e_{1}=\underset{t⟶\infty }{\lim}e_{2}=0. \end{array}$$

Above all, the adaptive kinematics model is used to design the sports rehabilitation; the control convergence and global stability are improved.

Through the above-mentioned design, the algorithm of the optimized control model of the lower extremity exoskeleton rehabilitation robot using the Lyapunov method and the inversion technique adaptive nonlinear tracking is obtained as follows.

Robot optimization control model algorithm:

1.  RRT.SetSConfig (***θ***_start_)//Set initial position
2.  do {//Perform a single tree RRT exercise planning cycle
3.   NormalExtend = true//Set random expansion tags
4.   *f*r = rand () ^*∗*^1.0/(0x7fff)//Generate 0∼1 random sampling probability
5.   if (*f*r≤*f* Extend){//Extension to body target pose
6.    NormalExtend = false//Indicates the expansion to the target pose
7.   ExtendStatus = **ExtendToGrasp** (RRT **p**_obj_**g**_*c*_)
8. if (ExtendStatus = = RRT_ERROR) {//Failed to expand
9.     StopSearch = true}//Set stop plan marker
10.    if (ExtendStatus = = RRT_REACHED){//Achieve goals
11. RRT.GetConfig **(*θ***_goal_**)**//Get the target configuration
12.      RRT.GetSolutionGrasp ()//Get the lower limbs bone movement goal solution
13.      FoundSolution = true**//**Search path solution}}
14.   if (NormalExtned) {//Random sampling configuration expansion
15.    RRT.RandomConfig (***θ***_rand_)**//**Generate random patterns
16.     ***θ***_near_ **=** RRT.NearestNeighbor (***θ***_rand_)//Recently shaped
17.    ExtendStatus **=** RRT.Connect (***θ***_near_,***θ***_rand_,***θ***_new_**)**
18. if (ExtendStatus = = RRT_ERROR){**//**Failed to expand StopSearch = true}}**//**Set stop plan marker
19.   Cycles++//Number of searches plus 1
20.  } while (!StopSearch && Cycles < MaxCycles && !FoundSolution)
21.  return RRT.GetSolutionPath (); }

## 4. Simulation Experiment and Result Analysis

In order to test the application performance of this method in the control of human exercise rehabilitation training, the simulation experiment is carried out. The hardware design part of the system selects ARM11 CPU as the central processor. Select ARM11 CPU S3 C6410 as the hardware core. DM9000 network card chip is used. DM9000 supports 8-bit, 16-bit, and 32-bit interface to access internal memory, and the design of control algorithm is taken. In this paper, the control parameter is selected as *λ*_1_=1, *λ*_2_=1, *c*_1_=2, *c*_2_=2, the initial value of parameter adaptive estimation is ${\hat{\delta }}_{0}=-15$, the adaptive parameter is *ε*_1_=0.1, and the human body is designed. The actual model parameters of sports rehabilitation training are as follows:

(33) $$\begin{array}{c} M_{p}=1.6\times 10^{4}\text{kg,}m_{r}=1.13\times 10^{4}\text{kg,}R=2.05\text{m},l=1.87\text{m,} \end{array}$$

(34) $$\begin{array}{c} K_{m}=0.0508\text{N.m}/\text{V}\text{,}K_{e}=0.5732{\text{V}}_{\text{s}}/\text{rad}, \end{array}$$

(35) $$\begin{array}{c} J_{p}=0.804\left(1\pm 0.5\right)\text{kg}\cdot {\text{m}}^{2},J_{r}=0.00623\left(1\pm 0.5\right)\text{kg}\cdot {\text{m}}^{2}. \end{array}$$

The state of the human skeleton is affected by many factors. In order to be closer to the actual situation, the subject must be allowed to walk in advance before the experiment is conducted, and the subject can start the experiment until it reaches a state of relaxation. As the human body walks, the left and right are basically symmetrical. This experiment only uses the right lower limb of the human body as the object of analysis.

Through experiments, the joints of the hips, knees, and ankles of the right leg can be measured with time and other motion information at different speeds. The hip angle refers to the angle between the thigh and the horizontal plane, and the knee angle refers to the lower leg. Between the thighs, the angle of the ankle refers to the angle between the foot support surface and the lower leg Taking a walking pace of 3.6 km/h as an example, after processing the data, the angle of each joint angle changes over time, as shown in Figure 3:

As you can see from Figure 3, the elevation angle of the robot's behavior in the assisted rehabilitation process is used as the evaluation index. The pitch tracking performance designed in this paper is shown in the figure. Using this algorithm, it has better robot control performance, and the control system can quickly track the input signal within 2 seconds without any control error. It has excellent anti-interference and robustness. Pitch elevation tracking of skeletal rehabilitation process is shown in Figure 4.

The human body model is mainly composed of muscles, bones, and ligaments. By introducing the acquired action capture data files into the AnyBody, the human walking motion can be simulated and analyzed by its walking simulation module. The simulation of the walking state is shown in Figure 5.

In the AnyBody simulation analysis, the kinematic analysis and the reverse dynamics analysis are used to obtain the kinematic information of the human body model and the information about the parameters of the muscles. The force of all muscles in the right leg during walking is obtained, as shown in Figure 6.

In the process of walking, not all bones are subjected to a large force. In order to study the force of the bones better and analyze the force of the muscles, only a part of the major muscles can be selected as the analysis object. From Figure 5, we can see that, in the course of walking in the last two cycles, the muscle force of the right leg peaked at 2.15s and 2.90s at two time nodes, respectively, and the muscle recruitment was larger at this time.

On the basis of the design of the simulation environment, the control system is designed to train the rehabilitation training of human body movement, and the visual recognition output of the body movement rehabilitation training is shown in Figure 7.

Figure 7 shows that the visual recognition ability of this method is good, and it has a good object-oriented ability. The control stability of human sports rehabilitation process is further tested, and the test results are obtained. Control performance test is shown in Figure 8.

As shown in Figure 8, the control system can track the input signal quickly within 2 seconds, and there is no control error at the same time. The control stability of this method is good for the rehabilitation training of human body movement.

## 5. Conclusions

This paper presents a design model of human motion rehabilitation based on object-oriented technology. The research contributions of the thesis mainly include the following aspects:

1. A visual dynamic tracking model for human movement rehabilitation is established.
2. Fuzzy PID superheterodyne control method is used to design the bone training control of human movement rehabilitation.
3. Bone tracking control and adaptive training are carried out under the control of object-oriented technology, and relevant data are collected for research.

Combined with object-oriented technology, the visual blur recognition of human sports rehabilitation training and the use of adaptive kinematics model to design the sports rehabilitation process can improve the control convergence and global stability of the human sports rehabilitation process. The simulation results show that the method has a good overall steady state and the sports rehabilitation training effect is obvious. This method has good application value in guiding sports rehabilitation training.

## Figures and Tables

**Figure 1:** Skeletal system modeling.

**Figure 2:** Exoskeletal structure after improvement.

**Figure 3:** Motion state setting of bone. (a) Hip joints. (b) Knee joint. (c) Ankle joint.

**Figure 4:** Pitch elevation tracking of skeletal rehabilitation process.

**Figure 5:** Walking state simulation.

**Figure 6:** All muscle force of human's right leg.

**Figure 7:** Visual recognition of human sports rehabilitation training based on object-oriented technology.

**Figure 8:** Control performance test. (a) Control simulation value of ankle joint rehabilitation training. (b) Control Simulation value of knee joint rehabilitation training.

## Data Availability

The data used to support the findings of this study are available from the corresponding author upon request.
